RETRACTED

# A Low-Power Stable Wideband Current Source for Acupuncture Point Skin Impedance Measurements

**DOI:** 10.1155/2021/6650651

**Published:** 2021-01-06

**Authors:** Changpei Qiu, Tianxia Zhao, Qiuping Li, Xin'an Wang, Kanglin Xiao, Bo Wang

**Affiliations:** The Key Laboratory of Integrated Microsystems, Peking University Shenzhen Graduate School, Shenzhen 518055, China

## Abstract

A low-power stable wideband current source for acupuncture point skin impedance measurements has been designed employing a differential architecture and negative feedback. The circuits extend bandwidth to 1 MHz, reducing harmonic distortion to 0.24% at 1 MHz. The output impedance is 37 MΩ at 100 kHz and 11 MΩ at 1 MHz. The stability of the output current of the current source when connected to different loads is below 0.1% at frequencies up to 500 kHz and increases to 0.74% at 1 MHz. The circuit was manufactured in a 0.13-*μ*m CMOS technology and measured results are presented. The area of the current source is 0.09 mm^2^ and its consumption is 1.2 mW. It is intended for low-power acupuncture point skin impedance measurements.

## 1. Introduction

Skin impedance measurement has been used for more than 50 years to measure changes in skin impedance at acupuncture points to help diagnose diseases and monitor the effectiveness of treatment [1, 2]. Over the years, researchers have used a wide variety of devices with many measurement modalities to measure skin electrical impedance. However, many interfering factors affect the validity of acupuncture skin impedance measurements. These factors include environmental conditions such as skin moisture, human physiological parameters, as well as the size and angle of the device used to measure skin impedance, the pressure of the measuring electrode, and the contact area with the acupuncture skin impedance [3]. The researchers point out that many of the possible sources of error in skin impedance measurements are related to the stability of skin impedance measurements. There are many methods [4, 5] for measuring skin impedance, including multichannel acquisition systems using concentric probes [6–8], as well as four-electrode and two-electrode probe methods [4, 7, 9]. However, the frequency variation of the injected skin current in these measurement methods and the variation of the system circuitry when intervening in the human skin impedance can affect the results of the skin impedance measurement. Skin impedance measurement typically uses a constant ac current source to inject current into the skin under test and then measure the voltage difference between the two sides of the skin to calculate the skin impedance. The current injection from the current source has to comply with the medical safety limits [10]. Skin impedance measurements can also be performed using an AC voltage source, where an AC voltage is injected into the skin to be measured, and the skin impedance is calculated by measuring the current signal through which it passes. This approach is used in biosensor applications [11–15]. However, voltage output biointerfaces are considered unsafe because when voltage is injected into the skin, the different skin impedances of different people cause different loads to the voltage source, and the resulting current cannot be controlled to a safe range, which can result in a higher risk of damage to different skin tissues [16].

RETRACTED

In skin impedance measurements, wideband operation is important. The ac current source must have a high accuracy bandwidth to prevent the output current of the current source from having large current errors due to variations in the cortical impedance load. The allowable injected current amplitude must comply with international safety standards [17]. As a result, the current source requires large output impedance in high-frequency broadband, and output current ensures low distortion and meets low-power requirements for acupuncture point skin impedance measurements which is limited in existing integrated current source [18–22]. For current source design studies, most have used the Howland topology circuit architecture, which is designed with discrete electronic component connections [22–25]. Current source design [24] uses a Howland topology to achieve a high output impedance (1.7 MΩ at 50 kHz) for the current source by using a resistor with a precision tolerance of 0.01%. However, in IC design, high precision resistors are difficult to guarantee. There are also current source designs that use a generalized impedance converter circuit to improve the output impedance of the current source by reducing the stray capacitance in the circuit [25]. The integrated current source proposed in [26] uses an active inductive load structure to implement an open-loop operational transduction amplifier (OTA), and its current source can reach an output impedance of 500 kΩ at 500 kHz, but the supply voltage is too high and the bandwidth is less than 1 MHz.

In this paper, we propose a low-power stable wideband current source for acupuncture point skin impedance measurements. The designed circuit uses the negative feedback technology formed by differential difference transconductance amplifier and output transconductance amplifier (DDTA-OTA) cascade with the on-chip sense resistors to improve the output impedance which ensures the stability of output current. The current source operates in 1.2 V power supplies and 40 *μ*A DC bias reducing power consumption. The paper is organized in the following sections.  Section 2 introduces the basic current source circuit and its linear current source architecture.  Section 3 focuses on the design of ICs for current sources. In Section 4 we perform performance tests on the current source circuits. In Section 5 we measured acupuncture point skin impedance. Finally, Section 6 concludes.

RETRACTED

## 2. Current Source Architecture

Figure 1 shows the basic current source circuit. *B* is the voltage buffer. The low frequency transfer function of the output current is

(1) $$\begin{array}{c} \frac{I}{V_{\text{in}}}=\frac{G_{m}}{\left(r_{0}+R_{L}+R_{S}\right)/r_{0}+R_{S}G_{m}}, \end{array}$$

where *G*_*m*_ is the OTA transconductance, *R*_*L*_ is the load resistance, *R*_*s*_ is sense resistors, *r*_0_ is the small-signal output resistance, *I* is the load current, and *V*_in_ is input AC voltage signal. For *r*_0_ ≫ *R*_*S*_+*R*_*L*_, the above expression simplifies to

(2) $$\begin{array}{c} \frac{I}{V_{\text{in}}}=\frac{G_{m}}{1+R_{S}G_{m}}\approx \frac{1}{R_{S}}. \end{array}$$

The current source circuit's output resistance is given by

(3) $$\begin{array}{c} R_{\text{out}}=r_{0}+\left(G_{m}r_{0}+1\right)R_{S}. \end{array}$$

If *G*_*m*_*R*_*S*_ ≫ 1, then *R*_out_ ≈ *G*_*m*_*r*_0_*R*_*s*_. Therefore, the use of negative feedback increases the output resistance of the circuit.

(4) $$\begin{array}{c} G_{m}=\frac{I_{\text{bias}}}{\left(V_{\text{GS}}-V_{\text{TH}}\right)}, \end{array}$$

where *V*_GS_ is the voltage across gate and source terminals of MOS transistor, *V*_TH_ is the threshold voltage, and *I*_bias_ is the DC bias current. The overdrive voltage of the transistor under SMIC 0.13 *μ*m CMOS technology is approximately 0.3 V. The permissible injection current amplitude must comply with international safety standards. For current frequencies less than 1 kHz where the load magnitude is 10 kΩ, the maximum allowable current flowing through the body is around 100 *μ*A [17], and when DC bias adopts 100 *μ*A and the sense resistor *R*_*S*_ is 500 Ω, *G*_*m*_*R*_*s*_ is far less than 1, so the effect of negative feedback increasing resistance is not produced.

### 2.1. Proposed Current Source Architecture

The current source structure consisting of preamplifier (DDTA_1_, DDTA_2_) and double-ended output transconductance amplifier (*Gm*_1_, *Gm*_2_) is shown in the block diagram of Figure 2. The AC voltage signal and the DC common-mode voltage are fed through the preamplifier to the next stage of the transimpedance amplifier to produce a stable output current. The output current is induced by the voltage across the integrated resistors and the generating voltage is fed back to the two-terminal input pair of the differential difference transconductance amplifier (DDTA_1_, DDTA_2_), thus establishing a negative feedback path.

RETRACTED

In the new current source, the voltage difference across the sense resistor is generated at the preamplifier (DDTA1, DDTA2), so there is no need to use a voltage buffer. The output current is generated by two current sources receiving a 180-phase shift differential input voltage signal (*V*in, −*V*in). Using the differential difference transconductance amplifier (DDTA) as the input stage can eliminate the unnecessary buffer parasitic added by the need for high-frequency operation and also isolate the load from the input signal. This current source structure expands the operating bandwidth and reduces the harmonic distortion of the output current, while also improving the output impedance of the circuit.

Assuming that the load is resistance *R*_*L*_, the low frequency transconductance of a single current source is given by the following equation:

(5) $$\begin{array}{c} G_{\text{current }}=\frac{I_{L}}{V_{\text{in}}}=\frac{1}{R_{S}+\left(\left(r_{0}+R_{S}+R_{L}\right)/r_{0}\right)\left(1/A_{\text{DDTA}}G_{m}\right)}, \end{array}$$

where *I*_*L*_ is the load current, *A*_DDTA_ is the small-signal voltage gain of the preamplifier, *r*_0_ is the small-signal output resistance, and *G*_*m*_ is the small-signal gain of the transconductor. The current source's output resistance is given by

(6) $$\begin{array}{c} R_{\text{out}}=r_{0}+\left(A_{\text{DDTA}}G_{m}r_{0}+1\right)R_{s}. \end{array}$$

The use of preamplifier (DDTA) can meet the condition that *A*_DDTA_*G*_*m*_*R*_*S*_ ≫ 1 by adjusting the gain of the preamplifier. Thus, *G*_current_ ≈ 1/*R*_*s*_. Hence, *G*_current_ can be set according to the value of the sense resistance, independent of the internal parameters of the circuit. The circuit structure of the negative feedback loop can enhance the output resistance of the current source circuit, thus eliminating the need to design a transconductor with a large output resistance. In the structure proposed in this paper, the output resistance of the overall circuit split in half because two current sources were connected in parallel to output current.

## 3. Current Source Circuit Design and Analysis

### 3.1. Preamplifier (DDTA)

In order to realize the negative feedback function of the whole circuit and further improve the output resistance, we designed a preamplification stage in this paper.  Figure 3 shows the COMS implementation of preamplifier in which a fully differential cascade to input differential difference pair formed by *M*_1_–*M*_4_. The *M*_1_–*M*_4_ transistors, as differential pairs, are connected to the *M*_11_–*M*_12_ as load diode to form the saturated MOS symmetrical load differential amplifier stage. Current mirrors consisting of transistor pairs *M*_15-16_*M*_13-14_ form a differential output stage with transistors *M*_19–22_.

RETRACTED

Common gate transistors *M*_17-_*M*_18_ provide active loading to the output differential pair. This circuit topology enhances the output resistance of the circuit and the gain of the differential output. The gate voltage of transistor *M*_10_ provides the DC bias for *M*_17-18_, which ensures that cascade pairs work in the saturation region. Transistors *M*_23_-*M*_24_ operate in the triode region and provide common-mode feedback (CMFB); they operate in the triode region. Cascade current mirrors formed by transistors *M*_5_–*M*_8_ provide the input bias current to the four-input differential difference pairs *M*_1_–*M*_4_. The advantage of this preamplifier topology is the ability to control the output stage of the circuit without affecting the input transconductance stage. The open-loop voltage gain of this circuit is given by

(7) $$\begin{array}{c} A_{\text{ov}}\approx G_{m}r_{\text{out}}\left[\left(V_{1}-V_{2}\right)-\left(V_{3}-V_{4}\right)\right], \end{array}$$

where *G*_*m*_ is the cross conductance in the whole circuit which is the product of the cross conductance of the input transistor and the gain of the current mirror (*G*_*m*_ ≈ *Bg*_*m*1_).

In order to provide sufficient bandwidth for the output current, we should ensure that the predominant pole frequency is large enough. Preamplifier circuit's internal node 1,2 is the low resistance node, while only output node 3 is the high resistance node. Main pole frequency *f* *d* is the −3 dB cut-off frequency:

(8) $$\begin{array}{c} f_{d}=\frac{1}{2\pi r_{\text{out}}\left(C_{n3}+C_{L}\right)}, \end{array}$$

where *C*_*L*_ is the parasitic capacitance of the input differential pair transistor of the next stage, *C*_*n*3_ is the parasitic capacitance of node 3, and *r*_out_ is the output impedance of node 3. To ensure sufficient phase margin, the nondominant pole must have a high enough frequency. The specific nondominant poles are generated at node 1, 4 and node 2, and the signals of node 4 and node 1 have the same amplitude and opposite phase, which constitute the nondominant poles of the full-differential signal. The frequencies of the nondominant poles generated in the preamplifier circuit are given by

(9) $$\begin{array}{c} f_{\text{nd}1,4}\approx \frac{g_{m1,4}}{2\pi C_{n1,4}}=\frac{g_{m1,4}}{2\pi \left(C_{\text{gs}16}+C_{\text{gs}15}+C_{\text{gs}11}\right)}, \end{array}$$

(10) $$\begin{array}{c} f_{\text{nd}2}\approx \frac{g_{m7}}{2\pi C_{n2}}=\frac{g_{m4}}{2\pi \left(C_{\text{gs}20}+C_{\text{gs}21}\right)}, \end{array}$$

where

(11) $$\begin{array}{c} C_{\text{gs}}=\frac{2}{3}C_{0x}\text{WL,} \end{array}$$

where *C*_ni_ is the parasitic node capacitance of ith node whereas *g*_mi_ and *C*_gsi_ are transconductance gain and gate to source capacitance of ith MOSFET. *C*_ox_ is the gate capacitance per unit area and *W* and *L* are the channel width and length of the devices.

RETRACTED

### 3.2. Transconductance Stage

Figure 4 is the schematic of the circuit of the transconductance stage. In order to improve the output impedance of transconductance stage, we adopted the common source common gate cascade technology and added the common gate transistor *M*_11_–*M*_18_. This circuit only has output node (*V*_out+_/*V*_out−_) which is high resistance node, and other nodes are low resistance nodes. Output impedance is made up of the resistance *r*_out13_ looking up from *M*_13_ and the resistance *R*_out17_ looking down from *M*_17_ in parallel given by

(12) $$\begin{array}{c} r_{\text{out}}=r_{\text{out}13}//r_{\text{out}17}, \end{array}$$

(13) $$\begin{array}{c} r_{\text{out}13}=r_{\text{ds}13}g_{m13}r_{\text{ds}8}, \end{array}$$

It can be seen that the adoption of the common gate transistor *M*_13_ and *M*_17_ increases *r*out_13_ and *r*out_17_ by rds.gm times. Perform the same procedures as before while ensuring adequate PMs and a single dominant pole. The single-ended output node current is the difference between the current supplied by the PMOS and NMOS transistors. The output current can be approximated by *I*_0_ ≈ *BG*_*m*_(*V*_1_ − *V*_2_) where *B* is the current mirror gain factor between *M*_5_ and *M*_7_, *M*_10_ (or *M*_6_ and *M*_8_, *M*_9_). The maximum output current amplitude allowed to be injected into the human body impedance must comply with international safety standards [17]. For AC signals injected into the human skin at a frequency of 1 kHz, the maximum allowable injection current amplitude for the human body is 100 *μ*A, and the maximum corresponding load is 10kΩ. In other words, the output voltage compliance is about 2 V. At output current frequencies above 25 kHz, the allowable current amplitude through the body is 2.5 mA, where the load magnitude is reduced to approximately 1 kΩ. We adopted low-supply-voltage (1.2 V) specification and the low-dc bias current (40 *μ*A), which can meet the high biological impedance load (100 kΩ) demand of human body and the maximum allowable load voltage of human body. The output voltage compliance of the OTA is

(14) $$\begin{array}{c} V_{\text{SS}}+V_{\text{ov}17}+V_{\text{ov}21}<V_{\text{out}}<V_{\text{DD}}-V_{\text{ov}8}-V_{\text{ov}13}, \end{array}$$

where *V*_SS_ and *V*_DD_ are negative power supply voltage and positive power supply voltages, *V*_ov*17*_ is the overdrive voltage of transistor *M*_17_, and *V*_ovi_ is the overdrive voltage of ith MOS transistor.

RETRACTED

To ensure low saturation voltage operation of the output transistors, OTA voltage compliance is designed to be ±1.2 V. When the outputs are short-circuited, the nominal gain of transconductance stage was designed for 144 *μ*A/V and the frequency of transconductance stage at a −3 dB bandwidth is approximately 10 MHz.

## 4. Current Source Circuit Measured Results

The proposed new current source was manufactured using a SMIC 0.13 *μ*m CMOS technology and can operate under 1.2 V power supply. Current source circuit is designed by Cadence software. The microphotograph of proposed circuit is shown in Figure 5. The area of the proposed current source is 0.09 mm^2^ and its power consumption is 1.2 mW. The on-chip sense resistors were chosen to be 500 Ω.

In order to eliminate the chance of measuring the performance of a current source circuit, five current source circuit chips were tested, each packaged on a designed pcb test circuit board. Pcb test circuit boards provide the necessary bias current and input/output signals for the current source chips. The chip was tested for the variation of the transconductance stage of the current source over the desired input AC voltage range, the accuracy of the output current of the current source in the frequency range 10 kHz to 1 MHz, and the distortion rate and output impedance of the output current of the current source chip.

The THD of the current source was evaluated using an Agilent E4411 B spectrum analyzer at 1 MHz. For three different input voltage amplitudes, corresponding to 50 *μ*A, 100 *μ*A, and 200 *μ*A output current amplitudes, the power of the output current harmonic frequency of the current source was measured 10 times at a time to measure the THD results. The measured THD was 0.1% for 50 *μ*A, 0.19% for 100 *μ*A, and 0.24% for 200 *μ*A.

Figure 6 shows the measurement results of the transconductance of the five current source chips. The result of transconductance of the current source was measured at a load of 10kΩ||5 pF and an input AC voltage signal operating at 1 MHz. The Agilent 33250a signal generator generates the AC voltage signal to provide the input signal to the current source. The maximum input voltage signal measured during normal operation of the chip is ±50 mV, and the maximum output current produced by the current source is 200*μ*Ap-p. The average transconductance tested for all five current source chips was 3.95 mA/V, and the standard deviation of the measured transconductance was 0.06 mA/V, where the maximum and minimum transconductance deviations were ±1.51%.

RETRACTED

Figure 7 shows the measured results of variation of transconductances of input AC voltage and the accuracy of the output current over frequency with a load of 10 kΩ//5 pF. In the frequency range 1 kHz to 5 MHz the accuracy of current source output is approximately 0.01% for 56 *μ*A, 84 *μ*A, 168 *μ*A, and 200 *μ*A. Between the 500 kHz and 1 MHz the accuracy of current source output is approximately 0.6% for 56.2 *μ*A, 0.63% for 84 *μ*A, 0.63% for 168 *μ*A, and 1.1% for 200 *μ*A. Besides, the measured result of output impedance shown in Figure 8 is at 37MΩ up to 100 kHz and 11 MΩ up to 1 MHz which ensured the stability of output current.

Another important purpose of the chip test is to test and study the stability of the output current of the current source circuit under different loads.  Figure 9 shows the measured output current of 10 *μ*A, 50 *μ*A, 100 *μ*A, and 200 *μ*A for different load impedance at 1 MHz. In the load impedance rang of 500 Ω to 10 kΩ, the stability of the maximum output current is below 0.1% at 500 kHz increasing to 0.74% at 1 MHz, respectively. The variability of output current in all five chips tested was less than 1%.

The proposed current source is compared with other publications, as is shown in Table 1. In both bandwidth variations, the proposed current source has achieved the highest output impedance and low harmonic distortion. And the power consumption is the lowest in Table 1.

## 5. Acupuncture Point Skin Impedance Measurements

Install the current source on impedance measuring device to obtain the impedance characteristics of human meridian acupoints and nonacupoint tissue specimens. This test uses a current source chip to test the electrical impedance of the skin around the human acupuncture point PC4 Ximen and non-acupuncture point PC4 Ximen surrounding area. The test data were used to distinguish the difference in electrical impedance between the skin around PC4 and nonacupoint PC4 area. During the test, subjects were asked to sit in a chair in a resting position and was advised to rest for 5 minutes before the measurement. Before the measurement, we performed an alcohol wipe on the participant's acupuncture point PC4 Ximen. The participant remained seated in a resting position while the measurement was obtained. Two (1.6 mm in diameter) silver electrodes used to test the skin resistance of the acupuncture points. One end of the electrodes is connected to the chip output port for receiving current from the current source chip and the other end is in contact with the measured acupuncture point.

RETRACTED

An output current of 20*μ*A_pp_ with a variation of current in the frequency range of better than 0.3% amplitude was injected into both sides of the acupuncture points. The output current was varied from 5 Hz to 800 kHz by controlling the input voltage. The voltage values at both ends were measured and recorded. The impedance spectra of the acupuncture points and non-acupuncture points were calculated as shown in Figure 10. It could be seen that the impedance of PC4 Ximen point was obviously different from the impedance of the peripheral non-points. By comparing the data in Figure 10, it is clear that the impedance of the acupuncture points is consistently lower than that of the surrounding area points at all frequencies. This finding is consistent with the results measured at fixed frequencies in previous acupoint impedance studies [28, 29].

## 6. Conclusion

A low-power stable wideband current source for acupuncture point skin impedance measurements has been proposed. The circuits extend bandwidth to 1 MHz, reducing harmonic distortion to 0.24% at 1 MHz. The output impedance is 37 MΩ at 100 kHz and 11 MΩ at 1 MHz. The stability of the output current of the current source when connected to different loads is below 0.1% at frequencies up to 500 kHz and increases to 0.74% at 1 MHz. More importantly, its power consumption is 1.2 mW which is intended for acupuncture point skin impedance measurements.

## Figures and Tables

**Figure 1:** Basic current source circuit.

**Figure 2:** The current source circuit structure block diagram.

**Figure 3:** The schematic diagram of the preamplifier stage (DDTA).

**Figure 4:** The schematic diagram of the transconductance stage.

**Figure 5:** Microphotograph of proposed circuit.

**Figure 6:** Transconductance of current source versus.

**Figure 7:** Variation of transconductances.

**Figure 8:** Output impedance with frequency.

**Figure 9:** Output current for different load impedance at 1 MHz.

**Figure 10:** Impedances of PC4 Ximen acupuncture point and nonacupoint PC4 Ximen surrounding area.

**Table 1:** Measured performance and comparison.

Parameter	This work	[27]	[21]	[26]
Technology	130 nm	180 nm	180 nm	350 nm
Supply	1.2 V	1.8 V	1.5 V	5 V
Bandwidth	>1 MHz	100 Hz–100 kHz	90 kHz	10 kHz–1 MHz
THD	0.24% at 1 MHz	0.2% at 100 kHz	1% at 90 kHz	0.79%@500 *μ*A
Power	1.2 mW	7.08 mW	2 mW	>10 mW
Max.output current	200*μ*A_p-p_	400*μ*Α_p-p_	350*μ*A_p-p_	500*μ*Α_p-p_
Output impedance	11 MΩ at 1 MHz	100 kΩ at 100 kHz	560 kΩ at 90 kHz	500 kΩ at 500 kHz
Current stability	0.74% at 1 MHz	None	None	None

## Data Availability

No data were used to support this study.
